# D-Dimer-to-Albumin Ratio: A Novel Indicator to Predict Poor Outcomes in Patients with HBV-Associated Decompensated Cirrhosis

**DOI:** 10.1155/2022/9062383

**Published:** 2022-09-13

**Authors:** Lin Sun, PingPing Ding, WeiLin Mao, JianPing Wu

**Affiliations:** ^1^Department of Clinical Laboratory, Shengzhou People's Hospital, Shengzhou Branch of the First Affiliated Hospital of Zhejiang University, Shengzhou 312400, China; ^2^Department of Clinical Laboratory, The First Affiliated Hospital, College of Medicine, Zhejiang University, Hangzhou, Zhejiang 310003, China

## Abstract

**Background:**

The purpose of the present study was to investigate the impact of D-dimer-to-albumin ratio (DAR) on outcomes in patients with hepatitis B virus-associated decompensated cirrhosis (HBV-DeCi).

**Methods:**

A total of 172 HBV-DeCi patients were enrolled. Logistic regression was used to explore the association between DAR and 30-day mortality. The area under the receiver operating characteristic curve (AUC) was used to evaluate the performance of DAR for predicting mortality.

**Results:**

The 30-day mortality was 19.8%. DAR was clearly higher in the nonsurvivors compared with the survivors, and increasing DAR was associated with an increasing risk of death. DAR was independently associated with mortality and its AUC for mortality was equivalent to that for Model for End-Stage Liver Disease score.

**Conclusions:**

DAR may be a potential prognostic marker for mortality in HBV-DeCi patients.

## 1. Introduction

Cirrhosis is one of the major causes of mortality worldwide and accounts for approximately 1 million deaths each year [1]. Hepatitis B virus (HBV) infection is the leading cause of cirrhosis in China [2]. Cirrhosis can be classified into two stages, compensated and decompensated, according to whether the disease accompanied by complications such as variceal bleeding, ascites, and encephalopathy [3]. Decompensated cirrhosis (DeCi) patients have poor outcomes and an estimated 5-year mortality rate of 85% [4]. Although liver transplantation improves the survival of DeCi patients, it is not widely used in clinical settings because of the insufficient numbers of donors, substantial costs, and immunological responses after transplantation. Therefore, it is important to establish an objective, accurate, and simple prognostic model that can identify high-risk patients and help guide clinicians when adjusting treatment strategies.

D-dimer is a fibrin degradation product, and abnormal plasma D-dimer levels have been detected in patients with thromboembolic events [5, 6], myocardial infarction [7], infection [8], autoimmune diseases [9], and various carcinomas [10–13]. Recent studies further showed that elevated plasma D-dimer levels can predict poor prognosis in patients with liver diseases [14–16]. Meanwhile, serum albumin is a simple marker that reflects nutritional status, and several studies have demonstrated associations between low serum albumin levels and unfavorable outcomes in acutely ill patients [17–19]. Therefore, it can be hypothesized that the combination of D-dimer and albumin levels may provide an accurate and convenient prognostic indicator for certain clinical problems. Küçükceran et al. [20] recently investigated a novel parameter called D-dimer-to-albumin ratio (DAR) as a marker for prediction of poor outcomes in COVID-19 patients. They suggested that DAR is a more valuable than any other parameter for predicting mortality. However, as far as we know, no published article investigated the relationship between DAR and the prognosis of HBV-DeCi.

Herein, we present an observational study to elucidate whether DAR could serve as a potential effective marker for 30-day mortality in hospitalized patients with HBV-DeCi.

## 2. Materials and Methods

### 2.1. Patients

The present study consecutively recruited 224 HBV-DeCi patients who were admitted to our hospital from December 2019 to February 2021. DeCi was defined by the development of ascites, encephalopathy, jaundice, or hepatorenal syndrome [21]. We excluded patients with (1) underlying liver diseases (e.g., other viral hepatitis, autoimmune, alcohol-, or drug-related liver diseases), (2) tumors, (3) hematologic disorders, (4) incomplete data, and (5) elderly age (≥75 years).  Figure 1 shows a flow diagram for the 52 patients who were excluded and the 172 patients who were finally included in the study. Patients received antiviral therapy and supportive treatment after hospitalization. The primary outcome was survival at day 30.

### 2.2. Ethics Statement

The study was performed according to the Declaration of Helsinki, and the procedures were approved by the Ethics Committee of the Shengzhou People's Hospital and The First Affiliated Hospital of the Medical College at Zhejiang University in China (approval number: 2018[598]).

### 2.3. Data Collection

Demographic and laboratory values, including sex, age, total protein, albumin, alanine aminotransferase (ALT), aspartate aminotransferase (AST), total bilirubin, creatinine, international normalized ratio (INR), D-dimer level, platelet count, and 30-day outcome, were derived from the institutional database. Biochemical values were measured using a Hitachi 7600 analyzer (Hitachi, Tokyo, Japan). Hematological parameters were measured using a Sysmex XE-2100 analyzer (Sysmex, Kobe, Japan). The D-dimer and INR were measured with a Sysmex CA1500 full-automatic analyzer (Sysmex Corp, Hyogo, Japan). The normal plasma D-dimer level at our hospital laboratory is less than 0.170 mg/L fibrinogen equivalent units (FEU). DAR was calculated as D-dimer level (mg/L) divided by albumin level (g/dL). At baseline, liver disease severity was assessed using the Model for End-Stage Liver Disease (MELD) score [22].

### 2.4. Statistical Analysis

Statistical analyses were performed using SPSS version 23 or MedCalc version 11.5 software. Statistical significance was defined as *P* < 0.05. Variables were presented as median with interquartile range or number. The demographic and clinical characteristics were compared using the Mann–Whitney test or *χ*^2^ test as appropriate. The association between DAR and MELD score was evaluated by Spearman correlation analysis. Univariate and multivariate logistic regression analyses were performed to identify independent risk factors for mortality in HBV-DeCi patients. Receiver operating characteristic (ROC) curves were drawn, and the areas under the curves (AUCs) were calculated to compare the prognostic performances of individual parameters.

## 3. Results

### 3.1. Patient Characteristics

A total of 172 HBV-DeCi patients were included in the present retrospective study. The main clinical events for hospitalization were uncontrolled ascites in 135 patients (78.5%), variceal bleeding in 57 (33.1%), clinical jaundice in 86 (50.0%), hepatorenal syndrome in 16 (9.3%), and hepatic encephalopathy in 18 (10.5%). The median serum DAR was 0.73 (range, 0.28–1.20). DAR had a positive correlation with MELD score (Figure 2).

Thirty-four patients had died by 30 days after admission. The causes of death were liver failure (*n* = 7; 20.6%), hepatorenal syndrome (*n* = 10; 29.4%), variceal bleeding (*n* = 7; 20.6%), and hepatic encephalopathy (*n* = 10; 29.4%). We divided the patients into nonsurvivors (*n* = 34) and survivors (*n* = 138) (Table 1). There were no significant differences in total protein, ALT, AST, platelet count, age, and sex between the two groups. However, significant differences were observed between the two groups for serum albumin, MELD score, total bilirubin, creatinine, INR, DAR, and D-dimer level (all *P* < 0.05).

### 3.2. Factors Associated with Mortality

The factors associated with poor outcomes in the univariate analyses included MELD score, D-dimer, DAR, and serum albumin. In the multivariate analysis, DAR and MELD score remained associated with mortality (Table 2). ROC curve analyses were performed to assess the values of MELD score and DAR for predicting prognosis. Baseline MELD score had a cutoff value of 16.2, with sensitivity of 88.2% and specificity of 56.5%, while DAR had a cutoff value of 1.07, with sensitivity of 61.8% and specificity of 77.5%. DAR had an AUC of 0.745, which was comparable to that for MELD score (AUC = 0.797; *Z* = 1.015; *P* = 0.310) (Figure 3).

### 3.3. Clinical and Laboratory Findings Related to DAR

Based on the DAR cutoff value of 1.07 determined in the ROC curve analysis, the 172 participants were divided into a high DAR group (>1.07; *n* = 52) and a low DAR group (≤1.07; *n* = 120). The 30-day mortality rate was 40.4% (21/52) in the high DAR group, compared with 10.8% (13/120) in the low DAR group. The high DAR group also had lower albumin, higher MELD score, higher ALT, higher D-dimer, and higher INR than the low DAR group (Table 3).

## 4. Discussion

DeCi is a syndrome with a high risk of death, but prediction of its clinical outcomes is challenging. In the present cohort, 34 patients (19.8%) had died by 30 days after admission. This mortality rate was higher than the rates of approximately 10% found in previous studies involving cirrhosis patients [23–25]. The discrepancy may arise from differences in the etiology or pathophysiology of the liver diseases in the patients enrolled in the studies. In a previous review of 118 studies, the 1-year mortality of cirrhosis patients was found to vary greatly from 1% to 57% based on the complications involved [26]. To improve outcomes, it is vital to identify high-risk patients and carefully select the therapeutic interventions. The MELD score is one of the most widely used indices for hepatic disease severity and was previously shown to predict mortality in liver diseases [22, 27, 28]. The MELD score involves three objective parameters: total bilirubin, INR, and creatinine. However, it has some drawbacks. First, it does not incorporate some important factors (hepatic encephalopathy and systemic inflammation) that can affect the prognosis of patients [29]. Second, it requires complex calculations and is inconvenient for routine practice. The present study explored the impact of DAR on outcomes in HBV-DeCi patients. DAR was found to be markedly increased in the nonsurvivors compared with the survivors. Furthermore, DAR was identified as a surrogate predictor of 30-day mortality in the multivariate analysis, and DAR at admission had an equivalent prognostic value to the MELD score. However, DAR involves evaluation of only two common biomarkers and is more convenient to use than the MELD score. Moreover, a recent study showed that low HDL-C level had a significant correlation with poor survival in HBV-DeCi patients. Our study indicates that DAR can also be used to predict prognosis in these patients [30].

The mechanism for the association between elevated DAR and HBV-DeCi prognosis involves many factors and remains poorly understood. The present results showed that elevated DAR could be attributed to increased D-dimer and decreased albumin. In previous studies, increased D-dimer was detected in several severe diseases and was linked to unfavorable outcomes in critically ill patients [31, 32]. Recently, a large multicenter cohort study showed that increased D-dimer was independently linked to adverse outcomes in critically ill patients with COVID-19 and further indicated that elevated D-dimer may be a general biomarker of disease severity rather than reflecting a unique pathophysiology driving mortality [33]. In other words, increased D-dimer may indicate a hypercoagulation state, but initiation of therapeutic anticoagulation on detection of increased D-dimer may be too late to change the pathological process. Numerous studies have indicated that elevation of D-dimer may reflect an underlying hypercoagulable state or inflammatory process or may itself be pathogenic [34–37]. Another study proposed that increased D-dimer may be associated with the complex pathogenesis of liver diseases, and they suggested that D-dimer is not only an index of the activation of fibrinolysis, but can also indicate systemic inflammation [16]. Meanwhile, serum albumin is exclusively produced by the liver and can reflect liver function, an important indicator during assessment of liver synthetic function and hypoalbuminemia that accounts for increased mortality in cirrhosis patients [38, 39]. Although plasma D-dimer and serum albumin levels were both identified as predictors of mortality in univariate analyses, neither were identified as predictors of mortality in the multivariate analysis carried out in the present study. This may arise because DAR, as a ratio, is more stable than its individual parameters, which may be influenced by factors such as hydration level or specimen handling. The study also revealed a positive correlation between DAR and MELD score and showed that increasing DAR was correlated with increasing risk of death, suggesting that DAR is closely linked to disease severity and hepatic dysfunction. Thus, we propose that DAR may be useful for evaluation of prognosis in HBV-DeCi patients. Further research is required to elucidate the underlying mechanism.

## 5. Conclusions

In summary, the present study suggests that DAR is a useful adjunctive marker for prediction of prognosis in HBV-DeCi patients. DAR is simple to calculate and can be used for early identification of poor outcome groups. However, the present study was limited by its retrospective nature and small sample size. Therefore, more studies are necessary to validate the findings.

## Figures and Tables

**Figure 1:** Flow chart of the included participants.

**Figure 2:** Scatter plots illustrating the positive correlation between DAR and MELD score (*r* = 0.226, *P* = 0.003) in HBV-DeCi patients.

**Figure 3:** ROC curves showing the prognostic performances of DAR and MELD score for prediction of poor outcomes in HBV-DeCi patients.

**Table 1:** Comparisons of baseline characteristics between the survivors and the nonsurvivors.

	All patients (*n* = 172)	Non-survivors (*n* = 34)	Survivors (*n* = 138)	*P*
Gender (female/male)	30/142	9/25	21/117	0.195
Age (years)	50.0 (43.0-58.5)	49.5 (40.0-57.0)	50.0 (44.0-59.0)	0.890
Total protein (g/dL)	5.86 (5.37-6.29)	5.72 (5.27-6.30)	5.89 (5.43-6.29)	0.284
Albumin (g/dL)	3.00 (2.75-3.37)	2.89 (2.62-3.19)	3.02 (2.77-3.41)	0.042
ALT (U/L)	67.0 (29.5-204.0)	71.0 (38.0-237.0)	64.5 (29.0-182.0)	0.312
AST (U/L)	73.0 (41.0-151.5)	75.0 (48.0-182.0)	73.0 (40.0-129.0)	0.250
Serum creatinine (*μ*mol/L)	66.0 (57.5-79.0)	74.5 (58.0-120.0)	65.5 (57.0-75.0)	0.025
Total bilirubin (*μ*mol/L)	171.4 (40.5-340.4)	278.9 (131.0-422.6)	146.5 (35.0-332.9)	0.003
INR	1.52 (1.29-1.85)	1.96 (1.52-2.42)	1.47 (1.26-1.76)	<0.001
Platelet (×10^9^/L)	83.5 (54.5-118.0)	77.5 (63.0-130.0)	84.0 (53.0-115.0)	0.722
D-dimer (mg/L)	2.14 (0.89-3.79)	3.82 (2.18-6.18)	1.86 (0.82-3.01)	<0.001
DAR	0.73 (0.28-1.20)	1.33 (0.76-2.35)	0.66 (0.24-1.04)	<0.001
MELD score	16.8 (11.2-21.2)	21.7 (18.5-25.7)	14.8 (10.1-20.2)	<0.001

Data are expressed as number or median (interquartile range). Abbreviations: ALT: alanine aminotransferase; AST: aspartate aminotransferase; INR: international normalized ratio; DAR: D-dimer-to-albumin ratio; MELD: Model for End-Stage Liver Disease.

**Table 2:** Factors associated with mortality of HBV-DeCi patients identified by logistic regression analyses.

	Univariate			Multivariate		
	Odds ratio	95% CI	*P*	Odds ratio	95% CI	*P*
Albumin (g/dL)	0.915	0.842-0.995	0.037			
MELD score	1.239	1.137-1.349	<0.001	1.209	1.107-1.319	<0.001
D-dimer (mg/L)	1.533	1.271-1.850	<0.001			
Age (years)	0.999	0.967-1.032	0.949			
DAR	3.027	1.847-4.960	<0.001	2.433	1.417-4.177	0.001

Abbreviations: DAR: D-dimer-to-albumin ratio; MELD: Model for End-Stage Liver Disease.

**Table 3:** Clinical data according to DAR values.

	Low group (DAR >1.07, *n* = 52)	High group (DAR ≤1.07, *n* = 120)	*P*
Gender (female/male)	10/42	20/100	0.851
Age (years)	51.5 (44.0-57.5)	50.0 (42.0-59.0)	0.506
Total protein (g/dL)	5.89 (5.55-6.40)	5.83 (5.33-6.26)	0.146
Albumin (g/dL)	2.84 (2.40-3.10)	3.10 (2.86-3.48)	<0.001
ALT (U/L)	40.5 (30.0-143.5)	77.5 (29.0-223.0)	0.101
AST (U/L)	72.5 (45.0-128.5)	73.0 (41.0-155.5)	0.901
Total bilirubin (*μ*mol/L)	137.0 (50.5-333.2)	216.5 (39.0-347.0)	0.681
INR	1.69 (1.46-2.19)	1.45 (1.24-1.72)	<0.001
Serum creatinine (*μ*mol/L)	66.0 (57.0-94.5)	66.0 (57.5-78.0)	0.324
D-dimer (mg/L)	4.36 (3.82-6.12)	1.33 (0.64-2.20)	<0.001
Platelet (×10^9^/L)	82.5 (52.5-130.0)	83.5 (55.0-114.5)	0.899
MELD score	18.2 (14.5-23.3)	15.8 (10.4-20.6)	0.010
30-day mortality (yes/no)	21/31	13/107	<0.001

Data are expressed as number, or median (interquartile range). Abbreviations: ALT: alanine aminotransferase; AST: aspartate aminotransferase; DAR: D-dimer-to-albumin ratio; INR: international normalized ratio; MELD: Model for End-Stage Liver Disease.

## Data Availability

The data are available upon reasonable request.

## Abbreviations

ALT: Alanine aminotransferase
AST: Aspartate aminotransferase
AUCs: Areas under the curve
CI: Confidence interval
DAR: D-dimer-to-albumin
DeCi: Decompensated cirrhosis
HBV: Hepatitis B virus
INR: International normalized ratio
MELD score: Model for end-stage liver disease
ROC: Receiver operating characteristic.

## References

[1] Tsochatzis E. A., Bosch J., Burroughs A. K. (2014). Liver cirrhosis. *The Lancet*.

[2] Xiao J., Wang F., Wong N. K. (2019). Global liver disease burdens and research trends: analysis from a Chinese perspective. *Journal of Hepatology*.

[3] European Association for the Study of the Liver (2018). EASL Clinical Practice Guidelines for the management of patients with decompensated cirrhosis. *Journal of Hepatology*.

[4] Wang S. B., Wang J. H., Chen J., Giri R. K., Chen M. H. (2012). Natural history of liver cirrhosis in South China based on a large cohort study in one center: a follow-up study for up to 5 years in 920 patients. *Chinese Medical Journal*.

[5] Lowe G. D., Haverkate F., Thompson S. G. (1999). Prediction of deep vein thrombosis after elective hip replacement surgery by preoperative clinical and haemostatic variables: the ECAT DVT Study. European Concerted Action on Thrombosis. *Thrombosis and Haemostasis*.

[6] Kwietniak M., Al-Amawi T., Błaszkowski T., Sulżyc-Bielicka V., Kładny J. (2017). The usefulness of D-dimer in diagnosis and prediction of venous thromboembolism in patients with abdominal malignancy. *Polski Przeglad Chirurgiczny*.

[7] Zhang H., Qiu B., Zhang Y. (2018). The value of pre-infarction angina and plasma D-dimer in predicting no-reflow after primary percutaneous coronary intervention in ST-segment elevation acute myocardial infarction patients. *Medical Science Monitor*.

[8] Kinasewitz G. T., Yan S. B., Basson B. (2004). Universal changes in biomarkers of coagulation and inflammation occur in patients with severe sepsis, regardless of causative micro-organism [ISRCTN74215569]. *Critical Care*.

[9] Inoh M., Tokuda M., Kiuchi H., Kurata N., Takahara J. (1996). Evaluating systemic lupus erythematosus disease activity using molecular markers of hemostasis. *Arthritis and Rheumatism*.

[10] Liu L., Zhang X., Yan B. (2014). Elevated plasma d-dimer levels correlate with long term survival of gastric cancer patients. *PLoS One*.

[11] Kilic M., Yoldas O., Keskek M. (2008). Prognostic value of plasma D-dimer levels in patients with colorectal cancer. *Colorectal Disease*.

[12] Mego M., Zuo Z., Gao H. (2015). Circulating tumour cells are linked to plasma D-dimer levels in patients with metastatic breast cancer. *Thrombosis and Haemostasis*.

[13] Altiay G., Ciftci A., Demir M. (2007). High plasma D-dimer level is associated with decreased survival in patients with lung cancer. *Clinical Oncology*.

[14] Li Y., Qi X., Li H. (2017). D-dimer level for predicting the in-hospital mortality in liver cirrhosis: a retrospective study. *Experimental and Therapeutic Medicine*.

[15] Qi T., Zhu C., Lu G. (2019). Elevated D-dimer is associated with increased 28-day mortality in acute-on-chronic liver failure in China: a retrospective study. *BMC Gastroenterology*.

[16] Zhou J., Mao W., Shen L., Huang H. (2019). Plasma D-dimer as a novel biomarker for predicting poor outcomes in HBV-related decompensated cirrhosis. *Medicine*.

[17] Akirov A., Masri-Iraqi H., Atamna A., Shimon I. (2017). Low albumin levels are associated with mortality risk in hospitalized patients. *The American Journal of Medicine*.

[18] Mishra P. M., Uversky V. N., Nandi C. K. (2020). Serum albumin-mediated strategy for the effective targeting of SARS-CoV-2. *Medical Hypotheses*.

[19] Chojkier M. (2005). Inhibition of albumin synthesis in chronic diseases. *Journal of Clinical Gastroenterology*.

[20] Küçükceran K., Ayranci M. K., Girişgin A. S., Koçak S. (2021). Predictive value of D-dimer/albumin ratio and fibrinogen/albumin ratio for in-hospital mortality in patients with COVID-19. *International Journal of Clinical Practice*.

[21] Liaw Y. F., Tai D. I., Chu C. M., Chen T. J. (1988). The development of cirrhosis in patients with chronic type B hepatitis: a prospective study. *Hepatology*.

[22] Freeman R. B., Wiesner R. H., Harper A. (2002). Lewis Teperman for the UNOS/OPTN Liver Disease Severity Score, UNOS/OPTN Liver and Intestine, and UNOS/OPTN Pediatric Transplantation Committees. *Liver Transplantation*.

[23] Xavier S. A., Vilas-Boas R., Boal Carvalho P., Magalhães J. T., Marinho C. M., Cotter J. B. (2018). Assessment of prognostic performance of albumin-bilirubin, child-Pugh, and model for end-stage liver disease scores in patients with liver cirrhosis complicated with acute upper gastrointestinal bleeding. *European Journal of Gastroenterology & Hepatology*.

[24] Cheng X. P., Zhao J., Chen Y. (2016). Comparison of the ability of the PDD-ICG clearance test, CTP, MELD, and MELD-Na to predict short-term and medium-term mortality in patients with decompensated hepatitis B cirrhosis. *European Journal of Gastroenterology & Hepatology*.

[25] Peng Y., Qi X., Guo X. (2016). Child-Pugh versus MELD score for the assessment of prognosis in liver cirrhosis: a systematic review and meta-analysis of observational studies. *Medicine*.

[26] D’Amico G., Garcia-Tsao G., Pagliaro L. (2006). Natural history and prognostic indicators of survival in cirrhosis: a systematic review of 118 studies. *Journal of Hepatology*.

[27] Botta F., Giannini E., Romagnoli P. (2003). MELD scoring system is useful for predicting prognosis in patients with liver cirrhosis and is correlated with residual liver function: a European study. *Gut*.

[28] Kamath P. S., Wiesner R. H., Malinchoc M. (2001). A model to predict survival in patients with end-stage liver disease. *Hepatology*.

[29] Stewart C. A., Malinchoc M., Kim W. R., Kamath P. S. (2007). Hepatic encephalopathy as a predictor of survival in patients with end-stage liver disease. *Liver Transplantation*.

[30] He X., Liu X. Y., Peng S. Q., Han Z., Shen J. J., Cai M. (2021). Association of low high-density lipoprotein cholesterol levels with poor outcomes in hepatitis B-associated decompensated cirrhosis patients. *BioMed Research International*.

[31] Lu J., Wang X., Chen Q. (2016). D-dimer is a predictor of 28-day mortality in critically ill patients receiving continuous renal replacement therapy. *Archives of Medical Research*.

[32] Shorr A. F., Thomas S. J., Alkins S. A., Fitzpatrick T. M., Ling G. S. (2002). D-dimer correlates with proinflammatory cytokine levels and outcomes in critically ill patients. *Chest*.

[33] Short S. A. P., Gupta S., Brenner S. K. (2021). D-dimer and death in critically ill patients with coronavirus disease 2019. *Critical Care Medicine*.

[34] Favresse J., Lippi G., Roy P. M. (2018). D-dimer: preanalytical, analytical, postanalytical variables, and clinical applications. *Critical Reviews in Clinical Laboratory Sciences*.

[35] Levi M., Thachil J., Iba T., Levy J. H. (2020). Coagulation abnormalities and thrombosis in patients with COVID-19. *The Lancet Haematology*.

[36] Al-Samkari H., Karp Leaf R. S., Dzik W. H. (2020). COVID-19 and coagulation: bleeding and thrombotic manifestations of SARS-CoV-2 infection. *Blood*.

[37] Yang Y., Tang H. (2016). Aberrant coagulation causes a hyper-inflammatory response in severe influenza pneumonia. *Cellular & Molecular Immunology*.

[38] Bernardi M., Ricci C. S., Zaccherini G. (2014). Role of human albumin in the management of complications of liver cirrhosis. *Journal of Clinical and Experimental Hepatology*.

[39] Romanelli R. G., La Villa G., Barletta G. (2006). Long-term albumin infusion improves survival in patients with cirrhosis and ascites: an unblinded randomized trial. *Journal of Gastroenterology*.

